# Effect of Evidence-Based Diet Nursing on Intestinal Flora and Maternal and Infant Prognosis in Patients with Gestational Diabetes

**DOI:** 10.1155/2022/1241530

**Published:** 2022-09-01

**Authors:** Ying Jiang, Chunbo Qiu, Yuanping Wang, Bin He

**Affiliations:** ^1^The Affiliated Hospital of Medical School of Ningbo University, Ningbo 315000, China; ^2^Ningbo Charity Maternity Hospital, Ningbo 315000, China

## Abstract

**Background:**

Gestational diabetes mellitus (GDM) refers to the diabetes first discovered or occurring during pregnancy. The incidence of gestational diabetes in China is about 1%–5%, with an increasing trend in recent years.

**Objective:**

To observe the effect of evidence-based diet nursing on intestinal flora and maternal and infant prognosis in patients with gestational diabetes.

**Methods:**

One hundred and thirty patients with GDM admitted to our hospital from January 2020 to January 2022 were selected and divided into two groups according to the intervention method, with 65 cases in each group. The control group was given routine nursing plus diet nursing, while the observation group was given evidence-based nursing plus diet nursing. The changes of blood glucose index and intestinal flora before and after intervention in the two groups were detected, and the compliance behavior, pregnancy outcome, and perinatal outcome in the two groups were statistically analyzed.

**Results:**

After the intervention, the fasting blood glucose, 2 h postprandial blood glucose, and HbA1c in the two groups gradually decreased (*P* < 0.05). Further comparison between the groups showed that the fasting blood glucose, 2 h postprandial blood glucose, and HbA1c in the observation group were lower than those in the control group (*P* < 0.05). After intervention, the ratios of *Bifidobacterium*, *Lactobacillus*, and *Bifidobacterium* to *E. coli* in the two groups gradually increased (*P* < 0.05). Furthermore, comparison between the groups showed that the ratios of *Bifidobacterium*, *Lactobacillus*, and *Bifidobacterium* to *E. coli* in the observation group were higher than those in the control group (*P* < 0.05). The blood glucose rate, regular prenatal examination rate, and diet control rate of the observation group were 100.00%, 100.00%, and 95.38%, respectively, which were higher than 89.23%, 92.31%, and 84.62% of the control group, and the difference was significant (*P* < 0.05). The pregnancy infection rate and cesarean section rate in the observation group were 0.00% and 33.85%, respectively, which were lower than 6.15% and 60.00% in the control group, and the difference was significant (*P* < 0.05).The premature delivery rate and polyhydramnios rate in the observation group were 3.08% and 1.54%, respectively, which were not significantly different from 6.15% to 7.69% in the control group (*P* > 0.05). The rates of macrosomia, neonatal hypoglycemia, and neonatal hyperbilirubinemia in the observation group were 1.54%, 3.08%, and 9.23%, respectively, which were lower than those in the control group (10.77%, 13.85%, and 23.08%), and the differences were significant (*P* < 0.05). The fetal malformation rate and neonatal asphyxia rate in the observation group were 0.00% and 1.54%, respectively, which were not significantly different from 1.54% to 7.69% in the control group (*P* > 0.05).

**Conclusion:**

The application of evidence-based care combined with dietary care in GDM patients can improve intestinal flora, control blood glucose, improve patient compliance behavior, and improve maternal and infant outcomes.

## 1. Introduction

Gestational diabetes can cause polyhydramnios, intrauterine infection, ketoacidosis, macrosomia, abortion, premature delivery, malformation, stillbirth, and other maternal and infant complications, which attracted clinical attention [1–3]. Reasonable dietary control and exercise therapy can restore blood glucose to the normal range in most patients, which needs to be combined with glucose-lowering medication if necessary. Quality nursing intervention plays an important role in the management of gestational diabetes [4, 5].

Evidence-based nursing is an emerging nursing model that combines nursing experience and patients' desires by finding evidence-based evidence from the previous high-quality literature to develop appropriate nursing measures, including three stages: raising questions, obtaining evidence-based support, and evidence-based nursing practice [6]. At present, evidence-based nursing has been applied in various clinical fields and has certain effects in promoting disease rehabilitation and improving prognosis [6, 7]. In this study, we observed the effects of evidence-based care combined with dietary care on intestinal flora and maternal and infant outcomes in patients with GDM for reference, which are reported as follows.

### 1.1. Core Tips

Effective management of gestational diabetes helps to improve pregnancy outcomes, but the effect of conventional intervention mode is not ideal. In this study, we implemented evidence-based care for patients with gestational diabetes and found that evidence-based care combined with dietary care could improve gut flora, control blood glucose, increase patient compliance behavior, and improve maternal and infant outcomes in patients with gestational diabetes.

## 2. Data and Methods

### 2.1. General Information

A total of 130 patients with gestational diabetes admitted to our hospital (January 2020–January 2022) were selected, aged 22–35 years, with an average of (28.12 ± 3.02) years. The gestational age was 25–33 weeks, with an average of (29.86 ± 2.55) weeks. They were divided into two groups using simple randomization, and there were 65 cases in each group.

### 2.2. Inclusion and Exclusion Criteria

Inclusion criteria include the following: (1) those diagnosed with gestational diabetes by the OGTT test [8]; (2) those aged 18–35 years; (3) all were singleton pregnancies with spontaneous conception; (4) those without other pregnancy complications and history of high-risk pregnancy; (5) those who complete clinical data.

Exclusion criteria include the following: (1) those with abnormal blood glucose before pregnancy; (2) those with communication and impairment; (3) those with comorbid severe psychiatric disorders; (4) those with growth hormone deficiency or other significant endocrine disorders; (5) those with known congenital malformations or genetic defects in the fetus; (6) those with gastrointestinal disorders; (7) those with comorbid other severe physical disorders.

### 2.3. Methods

The control group was given routine nursing plus diet nursing, and the body weight, blood pressure, and blood glucose were measured regularly for diet and exercise guidance. Patients who did not control blood glucose well in diet and exercise were given insulin therapy according to the doctor's advice, and the patients were guided to use insulin pen correctly. After 34 weeks of pregnancy, fetal heart rate and fetal movement were monitored regularly to evaluate the fetal intrauterine situation. Diet nursing: Dietary recipes were formulated according to the patient's blood sugar value, body weight, gestational age, and eating habits. The daily caloric intake of those with BMI less than 18.5 kg/m^2^ in the first trimester was 35 kcal/kg, the daily caloric intake of those with BMI of 18.5–23.9 kg/m^2^ was 30–35 kcal/kg, the daily caloric intake of those with BMI of 24.0–27.9 kg/m^2^ was 25–30 kcal/kg, the daily caloric intake of the BMI >28.0 kg/m^2^ was 30–35 kcal/kg, and the daily caloric intake of the second and third trimesters was increased 200–300 kcal on this basis. The proportion of carbohydrate, protein, and fat intake in the diet structure is 50–60%, 15–20%, and 20–30%. Pregnant women eat six times a day, and the calorie allocation for each meal is 10–15% for breakfast, 5–10% for breakfast, 30% for lunch, 5–10% for lunch, 30% for dinner, and 5–10% for dinner%.

The observation group was given evidence-based nursing plus dietary nursing. Dietary nursing was the same as that of the control group. Evidence-based nursing: an evidence-based nursing group was established with the head nurse as the team leader, and evidence-based nursing was implemented in three stages. (1) Asking questions: the following problems are found according to the problems found in daily nursing work, the needs of patients, and changes in the course of the disease: patients with gestational diabetes lack sufficient understanding of the harm of this disease; diet control cannot take into account the nutrition and health of pregnancy and blood sugar control; prone to negative emotions such as anxiety and depression; lack of exercise or improper exercise mode and exercise intensity; prone to gestational hypertension syndrome. (2) Obtain evidence-based support: we searched the CNKI database, Wanfang medical network, Chinese biomedical literature database, and so on according to the above questions. The keywords were GDM and nursing. We found evidence-based evidence and screened evidence according to nursing experience and course of disease through reading literature. (3) Evidence-based nursing practice: formulate an evidence-based nursing plan based on evidence-based evidence combined with nursing professional skills and experience. First, health education was provided to the patients to inform them of the hazards of gestational diabetes to the mother and baby and to instruct them to monitor blood glucose and count fetal movements correctly. Communicate and exchange with patients to understand the causes of negative emotions and use relaxation training and psychological suggestion to ease negative emotions. Instruct patients to exercise appropriately and develop individualized exercise programs, with aerobic exercise as the main focus. Blood pressure was measured regularly to detect and manage hypertensive syndrome during pregnancy in a timely manner. The nursing interventions in both the groups were carried out from the first visit to the delivery of the fetus.

### 2.4. Observation Indicators

The changes in blood glucose indexes and intestinal flora before and after intervention in the two groups were detected, and the medical compliance behaviors (adherence to blood glucose measurement, regular obstetric examination, and dietary control), pregnancy outcomes (preterm birth, polyhydramnios, infection during pregnancy, and mode of production), perinatal and neonatal outcomes (macrosomia, fetal malformation, neonatal asphyxia, neonatal hypoglycemia, and neonatal hyperbilirubinemia) of the 2 groups were counted.

### 2.5. Detection Method

Before and after the intervention, 2 ml of fasting venous blood was drawn from the patients in the morning, and the Beckman DXC800 biochemical analyzer was used to detect fasting blood glucose and HbA1c. Blood was drawn again 2 h after eating, and blood glucose was detected 2 h after meal in the same way.

The intestinal flora was detected before and after the intervention, and 0.5 g of the patient's fresh feces was added to sterile saline. The ATB semiautomatic microbial identification system of French BioMérieux was used to identify *Bifidobacterium*, *Escherichia coli*, and *Lactobacillus* and count the bifidobacteria/*Escherichia coli* ratio (B/E).

### 2.6. Statistical Methods

SPSS 19.0 was used to process the data, and the measurement indicators such as intestinal flora and dietary structure were first tested for normality, and those in line with the normal distribution were described by ($\bar{x}\pm s$), and the *t*-test was used for comparison. Those not in line with the normal distribution were described by median and quartiles, and the nonparametric test was used for comparison. The count data such as compliance behavior and pregnancy outcome were described by the number of cases (%) and compared by the *χ*^2^ test, and *P* < 0.05 was statistically significant.

## 3. Results

### 3.1. Comparison of General Data of Patients in the Two Groups

There was no significant difference in age, gestational age, pregnancy time, body mass index, maternal type, maternal occupation, total family income, education level, defecation frequency, and dietary structure between the two groups (*P* > 0.05), as given in Table 1.

### 3.2. Comparison of Blood Glucose Indexes between the Two Groups of Patients

The comparison between the groups before the intervention showed that the difference was not significant (*P* > 0.05). After intervention, the fasting blood glucose, 2 h postprandial blood glucose, and HbA1c of the two groups gradually decreased in the two groups (*P* < 0.05), and further comparison between the groups revealed that fasting blood glucose, 2 h postprandial blood glucose, and HbA1c in the observation group were lower than those in the control group (*P* < 0.05), as given in Table 2.

### 3.3. Comparison of Intestinal Flora between the Two Groups of Patients

The comparison between the groups before the intervention showed that the difference was not significant (*P* > 0.05). After intervention, the ratios of bifidobacteria, lactobacilli, and bifidobacteria to *Escherichia coli* in the two groups gradually increased in the two groups (*P* < 0.05), and further comparison between the groups revealed that the ratios of bifidobacteria, lactobacilli, and bifidobacteria to *Escherichia coli* were higher than those in the control group (*P* < 0.05), as given in Table 3.

### 3.4. Comparison of Medical Compliance Behavior between the Two Groups of Patients

The rate of adherence to blood sugar measurement, regular obstetric examination rate, and diet control rate in the observation group were 100.00%, 100.00%, and 95.38%, respectively, which were higher than 89.23%, 92.31%, and 84.62% in the control group, with significant differences (*P* < 0.05), as given in Table 4.

### 3.5. Comparison of Pregnancy Outcomes between the Two Groups of Patients

The infection rate during pregnancy and the cesarean section rate in the observation group were 0.00% and 33.85%, respectively, which were lower than 6.15% and 60.00% in the control group, with a significant difference (*P* < 0.05). The premature birth rate and polyhydramnios rate of the observation group were 3.08% and 1.54%, respectively, compared with 6.15% and 7.69% of the control group, and the difference was not significant (*P* > 0.05), as given in Table 5.

### 3.6. Comparison of Perinatal Outcomes between the Two Groups of Patients

The macrosomia rate, neonatal hypoglycemia rate, and neonatal hyperbilirubinemia rate in the observation group were 1.54%, 3.08%, and 9.23%, respectively, which were lower than 10.77%, 13.85%, and 23.08% in the control group, with significant differences (*P* < 0.05). The fetal malformation rate and neonatal asphyxia rate in the observation group were 0.00% and 1.54%, respectively, compared with 1.54% and 7.69% in the control group, and the difference was not significant (*P* > 0.05), as given in Table 6.

## 4. Discussion

GDM belongs to the category of high-risk pregnancy. It is a metabolic disorder caused by absolute or relative insulin deficiency and hyperglycemic secretion, the etiology of which is not completely clear. The existing research is based on multigene genetic defects, which is caused by pregnancy, obesity, stress, and other incentives [9–11]. GDM is more harmful and can increase the incidence of perinatal complications and mortality. Reasonable diet control can not only reduce insulin load and correct metabolic disorders but also prevent the failure of blood glucose control and hypoglycemia [12, 13]. Therefore, diet nursing is the basis and focus of nursing work for patients with gestational diabetes. The ideal gestational diabetes diet should not only meet the nutritional needs of pregnant women but also control fasting blood glucose, postprandial 2 h blood glucose, and nocturnal blood glucose in the normal range [14, 15]. However, in practical work, it is found that diet nursing alone often fails to achieve satisfactory nursing intervention effect [16, 17].

Evidence-based nursing is a more scientific nursing model and an important part of evidence-based medicine. In the process of planned nursing, the scientific research conclusions are combined with clinical experience and patient willingness to obtain evidence-based evidence as the basis for clinical nursing decision-making [18, 19]. In this study, evidence-based nursing was applied to the nursing of gestational diabetes, and it was found that the fasting blood glucose, postprandial 2 h blood glucose, and HbA1c of patients after intervention were lower than those of patients receiving routine nursing intervention (*P* < 0.05). The blood glucose rate, regular antenatal examination rate, and diet control rate of patients were higher than those of patients receiving routine nursing combined with diet nursing intervention (*P* < 0.05), suggesting that evidence-based nursing combined with diet nursing can improve the blood glucose control of patients with GDM and improve their compliance behavior. This is due to the fact that evidence-based care is guided by the problems found in the nursing work, the needs of patients, and the changes in the course of disease. It consults the literature, seeks, and filters evidence-based evidence and enables patients to realize the harm of gestational diabetes and the importance of a reasonable diet through health education, so that patients are more proactive in adhering to blood glucose measurement, regular antenatal examination, and dietary control [20, 21]. Through communication and exchange with patients, we understand that the causes of negative emotions and implement interventions to make patients cooperate with treatment in a more positive state of mind. Thus, patients are instructed to exercise appropriately, which is more helpful for blood glucose control [22, 23].

Intestinal flora is closely related to energy metabolism and abnormal of it can affect weight control and immune function [24, 25]. High glucose status in patients with gestational diabetes can alter the intestinal environment and cause changes in intestinal pH [26–28]. Probiotics such as *Bifidobacterium* and *Lactobacillus* are sensitive to changes in the internal environment, which can be significantly reduced once the intestinal environment changes [29–31]. While *Bifidobacterium* can regulate intestinal dysfunction, *Lactobacillus* can maintain intestinal health and regulate immune function, *Escherichia coli* is parasitic in the large intestine, and invasion of the body can cause infection. The ratio of *Bifidobacterium* to *Escherichia coli* can reflect the colonization of intestinal flora to some extent [32–34]. This study found that the ratio of intestinal *Bifidobacterium*, *Lactobacillus*, and *Bifidobacterium* to *Escherichia coli* in the patients receiving evidence-based nursing combined with diet nursing intervention was higher than that in the patients receiving routine nursing combined with diet nursing intervention, suggesting that evidence-based nursing combined with diet nursing can improve the intestinal flora of patients with gestational diabetes, which indirectly proves that evidence-based nursing combined with diet nursing is more conducive to blood glucose control.

Follow-up showed that the pregnancy infection rate, cesarean section rate, macrosomia rate, neonatal hypoglycemia rate, and neonatal hyperbilirubinemia rate of patients receiving evidence-based nursing combined with diet nursing intervention were lower than those receiving routine nursing combined with diet nursing intervention (*P* < 0.05). There was no significant difference in premature delivery rate, polyhydramnios rate, fetal malformation rate, and neonatal asphyxia rate between the two groups (*P* > 0.05), suggesting that evidence-based nursing combined with diet nursing can improve the maternal and infant outcomes of patients with GDM, which is related to the more stable blood glucose control of patients receiving evidence-based nursing intervention.

GDM can endanger maternal and infant health. Reasonable diet, exercise, medication, maintaining emotional stability, and preventing complications are the key points of intervention, but routine nursing and diet nursing cannot achieve satisfactory intervention effect. In this study, evidence-based nursing was used to intervene GDM on the basis of diet nursing. It was found that evidence-based nursing combined with diet nursing had greater advantages in controlling blood glucose, improving patient compliance behavior, and improving maternal and infant outcomes. This study further confirmed that evidence-based nursing combined with diet nursing can better improve the blood glucose level of patients with GDM by detecting the changes of intestinal flora before and after intervention.

In conclusion, the use of evidence-based care combined with dietary care in GDM patients can improve their intestinal flora, control their blood glucose, improve their compliance behavior, and improve their maternal and infant outcomes.

## Figures and Tables

**Table 1:** Comparison of general data of the two groups of patients.

Project		The control group (*n* = 65)	The observation group (*n* = 65)
Age (y)		28.56 ± 3.65	28.49 ± 3.25
Gestational week (week)		29.74 ± 2.15	29.83 ± 2.31
Pregnancy (second rate)		2.12 ± 0.53	2.18 ± 0.48
Body mass index (kg/m^2^)		28.45 ± 2.36	28.51 ± 2.42

Maternity type	Primipara	48 (73.85)	44 (67.69)
	Multiparous	17 (26.15)	21 (32.31)

Maternity occupation	Light stamina	40 (61.54)	41 (63.08)
	Medium stamina	25 (38.46)	24 (36.92)

Total household income (moon)	＜3000 yuan	11 (16.92)	8 (12.31)
	3000–6000 yuan	26 (40.00)	25 (38.46)
	＞6000 yuan	28 (43.08)	32 (49.23)

Educational level	Junior high school and below	7 (10.77)	6 (9.23)
	High school and college	38 (58.46)	37 (56.92)
	Undergraduate and above	20 (30.77)	22 (33.85)

Frequency of bowel movements (week)	≤2 second rate	0 (0.00)	0 (0.00)
	3–5 second rate	17 (26.15)	20 (30.77)
	6–7 second rate	42 (64.62)	39 (60.00)
	≥8 second rate	6 (9.23)	6 (9.23)

Diet	Dietary calorie intake (× 106 J/d)	4.45 ± 2.26	4.50 ± 2.31
	Percentage of protein intake (%)	19.02 ± 2.85	18.95 ± 3.01
	Carbohydrate intake percentage (%)	44.22 ± 8.23	43.98 ± 8.96
	Percentage of fat intake (%)	36.85 ± 5.23	37.02 ± 5.11
	Vegetable intake (g/d)	362.55 ± 75.26	354.11 ± 81.65

Compared with the control group, ^#^*P* < 0.05.

**Table 2:** Comparison of blood glucose indexes in the two groups of patients ($\bar{x}\pm s$).

Group	Number of cases	Fasting blood sugar (mmol/L)		2 h postprandial blood glucose (mmol/L)		HbA1c (%)	
		Before intervention	After intervention	Before intervention	After intervention	Before intervention	After intervention
The control group	65	9.25 ± 2.14	7.20 ± 1.45^*∗*^	11.85 ± 2.65	8.86 ± 2.11^*∗*^	12.25 ± 2.02	8.52 ± 1.45^*∗*^
The observation group	65	9.08 ± 2.36	6.65 ± 1.24^*∗*^^#^	11.81 ± 2.72	7.23 ± 1.54^*∗*^^#^	12.18 ± 2.25	7.02 ± 1.36^*∗*^^#^

Compared with the group before intervention, ^*∗*^*P* < 0.05; compared with the control group, ^#^*P* < 0.05.

**Table 3:** Comparison of intestinal flora between the two groups of patients ($\bar{x}\pm s$).

Group	Number of cases	*Bifidobacterium* (lgCFU/g)		*Lactobacillus* (lgCFU/g)		*Bifidobacterium* to *Escherichia coli* ratio	
		Before intervention	After intervention	Before intervention	After intervention	Before intervention	After intervention
The control group	65	6.25 ± 1.25	8.12 ± 1.36^*∗*^	5.36 ± 1.25	5.96 ± 1.28^*∗*^	0.72 ± 0.31	1.17 ± 0.34^*∗*^
The observation group	65	6.31 ± 1.21	8.86 ± 1.41^*∗*^^#^	5.30 ± 1.36	6.43 ± 1.08^*∗*^^#^	0.70 ± 0.33	1.31 ± 0.28^*∗*^^#^

Compared with the group before intervention, ^*∗*^*P* < 0.05; compared with the control group, ^#^*P* < 0.05.

**Table 4:** Comparison of medical compliance behavior of the two groups of patients (*n*, *%*).

Group	Number of cases	Keep checking blood sugar	Regular obstetric inspection	Diet control
The control group	65	58 (89.23)	60 (92.31)	55 (84.62)
The observation group	65	65 (100.00)^#^	65 (100.00)^#^	62 (95.38)^#^

Compared with the control group, ^#^*P* < 0.05.

**Table 5:** Comparison of pregnancy outcomes between the two groups of patients (*n*, *%*).

Group	Numberof cases	Premature birth	Polyhydramnios	Infection duringpregnancy	Ways to produce	
					Cesarean section	Vaginal birth
The control group	65	4 (6.15)	5 (7.69)	4 (6.15)	39 (60.00)	26 (40.00)
The observation group	65	2 (3.08)	1 (1.54)	0 (0.00)^#^	22 (33.85)^#^	43 (66.15)^#^

Compared with the control group, ^#^*P* < 0.05.

**Table 6:** Comparison of perinatal outcomes between the two groups of patients (*n*, %).

Group	Number of cases	Huge	Infant deformity	Neonatal asphyxia	Neonatal hypoglycemia	Neonatal hyperbilirubinemia
The control group	65	7 (10.77)	1 (1.54)	5 (7.69)	9 (13.85)	15 (23.08)
The observation group	65	1 (1.54)^#^	0 (0.00)	1 (1.54)	2 (3.08)^#^	6 (9.23)^#^

Compared with the control group, ^#^*P* < 0.05.

## Data Availability

The data used to support the findings of this study are available from the corresponding author upon request.
